The article "Technical Job Recommendation System Using APIs and Web Crawling" was published in 2022. Journal: Comput Intell Neurosci.

# Technical Job Recommendation System Using APIs and Web Crawling

**DOI:** 10.1155/2022/7797548

**Published:** 2022-06-21

**Authors:** Naresh Kumar, Manish Gupta, Deepak Sharma, Isaac Ofori

**Affiliations:** ^1^Department of Computer Science & Engineering, Maharaja Surajmal Institute of Technology, Janakpuri 110058, New Delhi, India; ^2^Department of Computer Science & Engineering, Moradabad Institute of Technology, Moradabad 244001, India; ^3^Department of Information Technology, Jagannath International Management School, Vasant Kunj, New Delhi 110070, India; ^4^Department of Environmental and Safety Engineering, University of Mines and Technology, Tarkwa, Ghana

## Abstract

There has been a sudden boom in the technical industry and an increase in the number of good startups. Keeping track of various appropriate job openings in top industry names has become increasingly troublesome. This leads to deadlines and hence important opportunities being missed. Through this research paper, the aim is to automate this process to eliminate this problem. To achieve this, Puppeteer and Representational State Transfer (REST) APIs for web crawling have been used. A hybrid system of Content-Based Filtering and Collaborative Filtering is implemented to recommend these jobs. The intention is to aggregate and recommend appropriate jobs to job seekers, especially in the engineering domain. The entire process of accessing numerous company websites hoping to find a relevant job opening listed on their career portals is simplified. The proposed recommendation system is tested on an array of test cases with a fully functioning user interface in the form of a web application. It has shown satisfactory results, outperforming the existing systems. It thus testifies to the agenda of quality over quantity.

## 1. Introduction

With an increasing number of cash-rich, stable, and promising technical companies/startups on the web [1] which are in much demand right now, many candidates want to apply and work for these companies. They tend to miss out on these postings because there is an ocean of existing systems that list millions of jobs which are generally not relevant at all to the users. There is an abundance of choices and not much streamlining. On the basis of the actual skills or interests of an individual, job seekers often find themselves unable to find the appropriate employment for themselves. This system, therefore, approaches the idea from a data point of view, emphasizing more on the quality of the data than the quantity.

### 1.1. Data Collection

The database used for this system was created using refined and customized data collection techniques and methods. This technique helps distinguish the database from the already existing commercially available job databases. Hence, data collection programs have been developed from scratch. Web crawling [2], as well as web scraping, has been used for dataset preparation. By combining web crawling and web scraping, more automation and less hassle were ensured on the Web with less human labor and error.

Different types of web crawlers used are as follows:

- Job Listing Crawler
- Ontology-based Crawler
- HTML Crawler
- API Crawler

### 1.2. Recommendation System

Recommendation systems proposed in [3] are mechanisms for information filtering that smartly identify and segregate information. They create smaller chunks out of large amounts of dynamically generated information. A recommendation system has the ability to predict whether a specific user will prefer an article or not based on their profile and its past information [4].

Collaborative filtering [5] makes recommendations based on historical user behavior. The model can only be shaped based on the behavior of a single user, as well as the behavior of other individuals who have used the system before them. Recommendations are based on direct collaboration from multiple users and then filtered to match those who express similar preferences or interests. Content-Based recommendations are specific to a specific user, as the model does not use any information about other users on the page.

#### 1.2.1. Content-Based Filtering

Content-based Filtering [6] is a machine learning technique that makes decisions by taking into account the similarities in the features of the data present. Two methods used to decide are as follows:

- Firstly, users provide a list of features out of which they can choose whatever they find the best.
- Secondly, the algorithm can keep track of the products that the user has shown interest in the past. They are appended to the users' already existing data.
- Content-based filtering recommenders do not need the profiles of other users or any foreign data as they do not greatly influence recommendations [7].
- *Collaborative Filtering.* The collaborative filtering method is based on the historical interlinkages that are documented among the users and items. The method tries to forecast the usefulness of articles for a specific user on the articles previously evaluated by fellow users. These memory-based methods work directly with the recorded interaction values and are based on finding the nearest neighbor, for example, finding the closest user of interest and suggesting the most popular product.

## 2. Related Work

In recent years, tremendous research has been done on the topic of job recommendations. For the completion of this paper, several research articles have been referenced which were published recently. With the help of this literature survey, it was seen that the basic steps involved in most of these recommendation systems are as follows:

- Data acquisition
- Data preprocessing
- Record recommendation

While several research papers and existing papers gave numerous insights on the problem statement at hand, all of them had some of the other elements of such a successful job recommendation system being in place: creating a scraping template: need to define HTML documents of those websites from where data needs to be collected; site navigation traversal: preparing a system for website navigation and exploration; automating navigation and extraction: conducting automation for the facts and processed data collected: computing data and packages from the website. The data acquired has to be saved in tables and databases.

The authors of [1], however, only focus on job aggregation and not filtering. One more limitation of [1] is that it relies only on HTML scraping to crawl the job listings, which does not always work in modern web applications due to client-side rendering of ReactJS, etc. They propose classification using Naïve Bayes on search engines. A web crawler is used to crawl individual company websites where the jobs are listed. For profile matching, they use two methods of matching: semantic similarity, tree knowledge matching, and query similarity. These are integrated based on the representation of attributes by students and companies; then the similarity is evaluated [2]. Kethavarapu et al. proposed an automatic ontology with a metric to measure similarity (Jaccard Index) and devise a reranking method. The raw data after collection goes through preprocessing. The process of ontology creation and mapping is done by calculating various data points to derive alternative semantics, which is needed to create a mapping. The module dealing with feature extraction is based on TF-IDF similarity and then the indexing and ranking of information by RF algorithm. The ranking/listing is achieved by the semantic similarity metric [3]. The authors of [4] focus on content-based filtering and examining existing career recommender systems. The disadvantages are the cold start, scalability, and low behavior. Its process starts with cleaning and building the database and obtaining data attributes. Then, the cosine similarity function is used to find the correlation between the previous user and the available list.

Mishra and Rathi give immense knowledge of the application domain accuracy measure and have finally compared them all. However, they use third-party aggregators to fetch the jobs and it is well known that these existing aggregators are not always updated. They cannot fetch jobs directly from the company portals [5]. Mhamdi et al. have designed/devised a job recommendation product that aims to extract meaningful data from job postings on portals. They use text accumulating methods. Resultantly, job offers are divided into job groups or clubs based on common features among them. Jobs are matched to job finders based on their actions [6]. The authors of [7] designed and implemented a recommender system for online job searching by contrasting user and item-based collaborative filtering algorithms. They use Log similarity, Tanimoto coefficient, City block distance, and cosine similarity as methods of calculating similarity. Indira and Rathika in their paper draw a comparison between interaction and accessibility of modern applications toward present conditions and the trustworthiness of E-Recruitment. The statistical tools used are Simple Percentage, Chi-square, Correlation, Regression, and ANOVA (One-way ANOVA) [8]. Pradhan et al. reveal a comparison between exploring relations amid known features and things describing items [9]. A system to make the proper recommendations based on candidates' profile matching as well as saving candidates' job preferences has been proposed in [10]. Here, mining is done for the rules predicting the general activities. Then, recommendations are made to the target candidate based on content-based matching and candidate preferences [10]. Manjare et al. proposed a specific model (CBF or content-based filtering) and social interaction to increase the relevance of job recommendations. Research exhibits high levels of management and flexibility [11]. In [12], matching and collaborative filtering were used for providing recommendations. They make a comparison of profile data and take a scoring in order to rank candidates in the matching technique. Consequently, the score ranking made recruiter decisions easier and more flexible. But since the scoring still had a few problems with coinciding candidate scores, a collaborative filtering method was used to overcome it.

The authors of [13] take a different spin on the topic by using modern ML and/or DMBI techniques in a RESTful Web application. They filled the difference between the Backend (MongoDB instance) and Frontend (Android Application) using APIs. An item-based collaborative filtering method for making job recommendations is presented in [14]. They optimized the algorithm by combining resume information and position descriptions. For optimizing the job preference prediction formula, historical delivery weight is determined by position descriptions. Similar user weight is computed from resume information [14, 15]. A system of web scraping for automatic data collection from the web using markup HTML and XHTML (classical markup languages) has been presented in [1]. The module of web scraping technique used by them was elucidated by four processes.

## 3. Proposed System

As we have seen, the present-day job seeker is faced with an array of problems before they can find a suitable job for themselves. All existing work is so promising but lacks in some of the other aspects. The need is to eliminate these issues posed by past research and minimize the weaknesses of the systems. The proposed system is designed to go forth with developing a fully functional user interface supporting a job aggregator and recommendation system. Every aspect of the operation is made from scratch and in a customized sort of manner.

Hence, the problem statement devised by us as a building starter for the research is as follows:

- Developing a hybrid model [16] that aggregates and recommends relevant jobs to the user based on their profile, skills, or interests.
- Emphasizing quality over quantity and delivering only the most appropriate results to the user. The results were achieved by applying intelligent filters and filtering out great amounts of data using appropriate parameters.
- Recommending jobs to users of any age and background in real time, based on the popularity of jobs among the other user base. Additionally, allowing users to study job popularity, skill demand, grossing market skills, etc. are discussed in [17, 18].
- Finally, designing a fully useable and understandable UI for the Recommender System for practical usage.
- The proposed system consists of the following three major modules, which are completed as part of this research as follows:
- Data collection and preprocessing [19, 20] followed by the unification of the database.
- Recommendation of suitable results using a hybrid system of content-based [21–23] and collaborative filtering.
- Development of a fully functional user interface in the form of a web application.

The flow diagram shown in Figure 1 is used as the proposed system architecture for the modeling process and demonstrates a high-level design of the entire aggregation and recommendation system. The modules of the proposed architecture have been used in the implementation.

### 3.1. Data Collection and Preprocessing

The data collection and preprocessing module was further divided into four submodules. All these modules depicting the different kinds of data needed to be collected as part of this research are categorized as follows.

#### 3.1.1. Company Fetching Module

This module is used to fetch and list the top N companies (we started with the top 100 companies) based on the rankings on platforms such as Crunch base [24]. To get the list of these companies automatically, the web crawler [25, 26] reads and parses the API calls of platforms. After parsing, this module converts the list into the form of a large JSON array with each element of the array being an object representing each company.

A superset of all potential companies is created. This ranking is not completely polished and further filtering is to be performed. Appropriately selected critical parameters are used to further enhance the quality of the database.

#### 3.1.2. Company Detail Gathering Module

This module is used to collect important deciding details about a particular company that will be used to filter the companies from the list. These parameters are important to shortlist only the best companies, so that irrelevant options are not displayed to the user. This was done by crawling and scraping the concerned web listings [27, 28] for these companies.

The parameters that have been used to filter out companies are series of funding, total funding, number of investors, number of employees (organization size), unicorn status [29], and latest technology stack.

Upon using these parameters, a new list of shortlisted companies has been created which has fewer results. This is the final list of this research and recommendation system [30] to work upon.

#### 3.1.3. Job Listing Fetching Module

This is a very critical module and its function is to scrape and crawl the respective sources for the job openings of the shortlisted companies and aggregate them in the database. For the course of this research paper, new and customized crawlers have been designed from scratch, instead of using third-party aggregators [31, 32]. Typically, all these common aggregators tend to miss out on the latest job listings and a major objective of this system is to remove this anomaly. The job listing fetching has been done using the following three types of crawling techniques.

#### 3.1.4. Job Listing Platform Crawling

Using this crawler, the crawling was initiated from a set of URLs [32, 33]. BFS technique [34] was used to further crawl the rest of the URLs.

#### 3.1.5. Standalone Company Website Crawling

Nowadays, many companies do not list their job openings on the common job listing portals on the web [35–49]. It was decided to individually crawl the API calls [50, 51] of these companies' personal job portals. Different companies had different kinds of embedding of the abovementioned job listing portals. Hence, a combination of many kinds of crawling techniques was used as follows:

(o) Ontology-based crawler is being based on the concept of ontology and only crawls pages related to a given/specific topic.
(o) API-based crawler is very useful since most of the web applications in today's age do not use simple HTML. It is required to make an API crawler that can intercept API calls of the career pages and fetch the required result.
(o) HTML crawling: a lot of older companies that were part of the final list of shortlisted companies still used HTML encoding. Hence, crawling of those company portals was done using HTML scraping. This is not a single crawler but a group of crawlers working in parallel, traditionally in the same network. This testifies the research that doing this improves the efficiency of the crawler by optimizing the speed.

#### 3.1.6. Data Fields Unifying Module

Data of various job postings, listed by various platforms as well as standalone companies' job portals, is collected. This was done after culminating a list of the companies that the paper was going to move ahead with, using various filters as mentioned in submodule C. This concluded the data collection part of the research. The job listings achieved as a result of the abovementioned data collection are, however, not uniform. There are irregularities in the data with respect to incoherent key-value sets used by various companies. They did not have a common schema [52].

For example, a company *X* might label their job description as “JD”, company Y could name the same information under “Details”, and company *Z* could name it as “Requirements”. With such incoherence and nonuniformity, the database cannot be directly used for further tasks. It was, hence, unified.

A procedure was devised for the one-time unification of the database for each company [53]. It can then be reused for all job listings from that company in the future. For each company, however, this unification needs to be done at least once. All fields related to the kind of role were unified and named “Title”, all fields of job description and requirements were filed under “Description”, etc. A total of nine such headers or keys were unified. The schema thus obtained looked like this:

Schema({
    job_id: String,
    title: String,
    description: String,
    location: String,
    company: String,
    platform: String,
    apply_url: String,
    created_at: String,
    updated_at: String
});

As a result of this, the unified database with a common schema is now ready to be used by the filtering algorithm.

### 3.2. Recommendation System

Now, the data aggregation and collection part has been implemented, and the data has been unified in the database. It is ready to be used to recommend jobs to the user. The proposed system calls for a hybrid system of content-based and collaborative filtering. The system contrasts this particular hybrid method with the two types of filtering used individually to see how the hybrid system delivers results. These results are more practically visualized in the web application when the recommendations are listed for the user.

(1) Content-based filtering finally provides the recommendation of the list of appropriately matching jobs. It is implemented in two ways:
  - *Profile-Description Matching.* In this functionality, the user can be recommended for jobs on the basis of the user profile that they have fed to the portal. Using a host of algorithms, the user profile is matched against the unified job listing database previously created.
  - *Keyword-Based Searching.* In this functionality, jobs will be recommended on the basis of explicit searching by the user. The user will be able to enter the keywords, their skills, interests, or job areas they are interested in. The system will recommend jobs after matching those particular keywords with the job descriptions of companies.

The jobs are listed in the decreasing order of appropriateness to the user. It is unique for each user based on their profile. Both of these functionalities are achieved through content-based filtering cum CBF. It attributes to recommend another similar item that the user likes, based on their past actions or clear feedback. User profiles are built using existing actions or by explicitly asking users about their preferences. For new users, the latter is a more proper technique. As the system gets trained over time, the model will learn to recommend the jobs that the user previously showed interest in. This hypothesizes the fact that if a user is interested in a particular job category, they will be interested in something similar in the future. It is true as the skillset of a jobseeker remains more or less static over time. However, there can always be room for new additions to their profiles. As mentioned, for new users, explicitly taking an input of their interests or skills or requirements is the best way to move forward.

#### 3.2.1. Content-Based Filtering Algorithm

After the recommender is trained by an array of documents, it can tell the list of documents that are more similar to the input document. The training process involves three main steps as follows:

- Content preprocessing is used to clean all job descriptions and user profiles by removing and eliminating all the common English connectors and conjunctions. These are known as ‘stop words'. These can be ‘and', ‘can', ‘but', ‘is', ‘has', etc. In addition to this, it also removed HTML tags that are present in the descriptions due to HTML scraping. This is known as HTML tag stripping.
- It computes document vectors using the concepts of Term Frequency (TF) and Inverse Document Frequency (IDF). It gives the count of occurrences of the input term in the entire document domain.
- Cosine similarity is one of the important elements of content filtering. This similarity is calculated between all vectors in the document.

TF and IDF concepts are used to assess the relative value of documents, articles, or works. The count of the word in a document is measured in TF. The recurrence of all documents is the IDF. The effect of high-frequency repetitions in evaluating the exclusion of an object is rejected by the TF-IDF. However, the mathematical tool log is used to minimize the impact of any repetitive words when calculating the TF-IDF.

The significance of the word in a document cannot be determined by a simple raw number. It leads to the following :

(1) $$\begin{array}{c} w_{t,d}=1+{\text{log}}_{10}tf_{t,d}tf_{t,d}>0,\\ w_{t,d}=0\text{otherwise},\\ tf_{t,d}⟶w_{t,d},\\ 0⟶0,1⟶1,2⟶1.3,10⟶2,1000⟶4. \end{array}$$

(o) *Cosine Similarity.* For two N-dimensional vectors' cosine values, cosine similarity indicates the degree of similarity between the vectors. The higher the values of cosine similarity, the closer the two document vectors in question in similarity. This value is typically between 0 and 1 since there are no negative vectors. Equation 2 is used to calculate the cosine.

(2) $$\begin{array}{c} S\left(Q,D\right)=\frac{\in Q_{w}.D_{w}}{\sqrt{\in Q_{w}^{2}.D_{w}^{2}}}, \end{array}$$

where *S* is the similarity value, *Q* is the document vector 1, and *D* is the document vector 2.

What the model does for new users is that it matches the user's profile with the job description listed by the company in their respective job postings. It parses all job descriptions, looking for matches suitable for the user's profile. Based on these matchings, a match percentage or a match score is calculated. Using this score, job listings are displayed to the user in descending order of their match percentage.

This module has been tested on a fair number of test cases and has shown satisfactory results every time. Each test case was catered to mimic the behavior of a different user, each having a separate set of skills and interests.

#### 3.2.2. Collaborative Filtering:

In collaborative filtering, the idea is to find similar users and recommend to each one of them what users similar to them like. In this sort of recommendation system, instead of using the features of the item to make recommendations, classification of the users into clusters of analogous types is done. The system recommends each user on the basis of the preference of its respective cluster.

There are two types of collaborative filtering methods: (i) user-based approach and (ii) item-based approach.

In the user-based approach, the users are the masters of the ring. If some users have a similar preference, they tend to join a group. Recommendations are given to the user, built on the evaluation of items by other users in the same group. These users share a common taste. The reason for such a filter being chosen in the paper is that the prediction is mainly based on the average weight of recommendations from many people. It is located in a single bank from the same person. The weight allocated to the individual assessment determines the relationship between the user and the other user. Pearson's correlation coefficient was used to measure this correlation.

*(1) Pearson Correlation Coefficient*. This correlation method was used to compute how much the similarity of mutual users for particularly two items deviates from the average ratings. The range of the Pearson coefficient varies between the values zero and one. The larger the magnitude of this coefficient, the higher the correlation between the two documents. It is depicted in the following equation:

(3) $$\begin{array}{c} P=\frac{n\left(\in ab\right)-\left(\in a\right)\left(\in b\right)}{\sqrt{\left(\left[n\in a^{2}-\left(\in a^{2}\right)\right].\left[n\in b^{2}-\left(\in b^{2}\right)\right]\right)}}, \end{array}$$

where *P* is the Pearson coefficient, and *a* and *b* are two entities.

Talking about the implementation of collaborative filtering, the system generates recommendations for a user based on users with a similar taste. There is no normalization based on popularity at the moment, hence, no room for any bias depending on the user profile.

Another important assumption made is that the system is not taking into account any dislikings or spam jobs. In other words, the paper takes into account the jobs only which have been recommended by similar users. An array matrix is defined which is an *M* ∗ *N* matrix with *M* being the number of users and N being the jobs. The engine defines the ratings of the users in the database. It contains only Boolean values: 0 (not rated) or 1 (recommended or applied). After the function gets the required input in the above format, it runs through the collaborative filter algorithm. The algorithm effectively generates job recommendations using Jaccard Similarity.

*(2) Tanimoto Coefficient (Jaccard Index)*. The Jaccard Similarity Index or Tanimoto coefficient is a degree of similarity between two sample sets of data. The index arrays are from 0 to 1. The closer to 1, the more similar are the two data sets.

Jaccard Similarity = (Intersection of the two sets of the number of observations common in both sets)/(Union of the two sets or the number in either of the sets).

Equation (4) is a mathematical representation:

(4) $$\begin{array}{c} J\left(A,B\right)=\frac{A\cap B}{A\cup B}. \end{array}$$

Using this concept, a methodology for computing similar jobs based on collaborative filtering [53, 54] is devised. Some machine learning algorithms can also be devised [55]. The system first finds similar users (who have applied to the job) and the jobs to which these common users have applied. Based on the correlation and similarity between the two users, jobs will be recommended to the current user. That means a job applied by User 2 would be recommended higher than the one applied by User 3 if User 1 is more similar to User 2 than User 3.

#### 3.2.3. Hybrid Recommendation System

The concept of a hybrid recommendation system is based on the fact that content-based and collaborative filtering alone does not provide the best job recommendations to the user. Therefore, a method to combine the two types of filtering and make the recommendation engine truly hybrid was devised. To achieve this, the system first finds similar users and jobs as discussed above in collaborative filtering. After this, the correlation score for the recommended job is computed. To calculate this, the ratio of the number of common jobs between the main and suggested user to the number of all common jobs present between all the users is taken. This way, a score between 0 and 1 is generated. Taking the average of the score computed just above the content-based filtering score, the system produces a final recommendation score for each job. This way, it is possible to rank all top-recommended jobs to the user based on a hybrid model of content-based and collaborative filtering.

## 4. Algorithm

Algorithmic steps for weight determination, content score, collaborative filtering, and hybrid score calculation are shown in Algorithm 1.

## 5. Results and Analysis

Table 1 shows the comparison between the standard existing job recommendation models in the market (naukri.com, indeed.com) and existing research papers. The following parameters were derived from it.

Table 2 summarizes the top seven jobs liked by some particular users in the system were analyzed and the content-based and hybrid scores for them were compared as shown in the table.

From Figure 2, it is observed that the average percentage increase in the match score is 59.78%. In content-based filtering, it was tried to recommend the jobs as per the user's profile and resume by parsing all job descriptions and computing a match score.

For this, two experiments were performed: one with the raw job description and the second after processing the jobs. The comparison between the two can be seen in Table 3.

Figure 3, clearly, shows that the average percentage time reduction after processing the descriptions is 37.74%.

Table 4 is an extension of the above experiment and a more important metric was observed, i.e., the match score. The input was the same as the above previous one.

Figure 4 shows that job description processing increases the chances of the user getting matched to his desired job by 103.44%.

## 6. Conclusion and Future Scope

In this paper, Content-Based Filtering and Collaborative Filtering of recommendations have been compared. Additionally, an aggregation plus recommender system has been devised. Content-Based Filtering recommends the results based on matching the personal preferences of the user with the given document whereas collaborative filtering recommends based on the preferences of fellow users. On evaluating both of these methods, it was concluded that a hybrid system of both of these overcomes the limitations of both of them and increases the efficiency of ranking. Problems of cold start, sparse database, scalability, and lack of trend recommendation [5] have been eliminated. The proposal is to design a Job Recommender system that prioritizes quality over quantity. While there are websites and job listing portals already recommending jobs to job seekers based on their profiles, this research on aggregate quality recommendations has been achieved by crawling selectively, overcoming the limitations of [1, 4, 14]. A fully functioning user interface was developed to combine everything together to give the user a seamless experience.

For this system to be hybrid, content-based filtering is required, which can only recommend jobs based on the user's current profile. It cannot deliver anything surprising based on the user's past searches. This paper also uses collaborative filtering which faces well-known problems of privacy breaches and cold start. The system has a broad scope that can be used to make it more robust and foolproof. Firstly, automating the crawling process is required, when a new company is added to the database. In other words, removing the one-time configuration step/process to fetch jobs of a particular new company can be done. These models can implement techniques such as KNN in collaborative filtering. Implementing NLP in content-based filtering for better and more accurate search matching can be done. Along with this, testing and collecting more user data for better performance of the collaborative filtering module is required. Lastly, improving the cleansing process of the job description and using natural language processing are required. While using collaborative filtering, this work can be improved by giving different weights to different users based on their LinkedIn skills.

## Figures and Tables

**Figure 1:** Proposed system architecture.

**Figure 2:** Comparing ranks of relevant jobs in content-based and hybrid recommendations.

**Figure 3:** Comparing the efficiency of the system with and without preprocessing the job descriptions.

**Figure 4:** Comparing ranks of jobs after preprocessing the descriptions.

**Algorithm 1:** Hybrid recommendation system.

**Table 1:** Comparing the features of existing systems with the proposed system.

Systems	Aspects			Companies listed		
	Data collection method	JD cleaning	Recommendation methodology	Real time	Jupiter	Pratilipi
Reference [2]	College campus	No	Content-based filtering	No	NA	NA
Reference [25]	Single website crawler	Yes	No	No	No	No
Naukri	Direct listing	Yes	Collaborative	No	No	Yes
Indeed	Direct listing	No	Collaborative	No	No	No
Proposed system	Automate crawling	Yes	Hybrid system	Yes	Yes	Yes

**Table 2:** Comparing ranks of relevant jobs in content-based and hybrid recommendations.

Job_ID	Rank before (content)	Rank after (hybrid)
61a29356c062e596f369e488	9	1
61a293c9c062e596f369e6ad	5	2
61a293c6c062e596f369e6a1	20	3
61a2936dc062e596f369e4f4	6	4
61a29357c062e596f369e491	1	5
61a293c7c062e596f369e6a4	3	6
61a2936dc062e596f369e4f7	19	7

**Table 3:** Comparison of the efficiency of the system with and without preprocessing the job descriptions

User skills/description	Time taken for the raw job description (s)	Time taken for the processed job description (s)	Percentage reduction in time (%)
Test case 1—frontend	33.38	20.87	37.48
Test case 2—backend	29.54	19.55	33.82
Test case 3—machine learning	51.07	36.69	28.16
Test case 4—DevOps	46.28	29.52	36.21
Test case 5—product management	38.48	18.07	53.04

**Table 4:** Comparing the ranks of jobs after preprocessing descriptions.

User skills/description	Average match score for raw job description	Average match score for processed job description	Percentage increase in the match score (%)
Test case 1—frontend	0.05629	0.12358	119.54
Test case—2 backend	0.04631	0.09131	97.17
Test case—3 ML	0.04672	0.10409	122.8
Test case—4 DevOps	0.06277	0.11382	81.33
Test case—5 product management	0.22237	0.45107	102.85

## Data Availability

The data used to support the findings of this study are available from the corresponding author upon request.
